The article "Overexpression of miR-499-5p inhibits non-small cell lung cancer proliferation and metastasis by targeting VAV3" was retracted in 2021. Reasons: duplicated images; original data or images not available; unreliable data; concerns about the data.

# Overexpression of miR-499-5p inhibits non-small cell lung cancer proliferation and metastasis by targeting VAV3

**DOI:** 10.1038/srep23100

**Published:** 2016-03-14

**Authors:** Ming Li, Shenjun Zhang, Ning Wu, Liang Wu, Changhui Wang, Yinping Lin

**Affiliations:** 1 Department of Respiratory Medicine, Shanghai 10th People’s Hospital, Tongji University, Shanghai 200072, China; 2 Institute of Biochemistry and Biology, Shanghai Institutes for Biological Sciences, Chinese Academy of Sciences, Shanghai 200031, China; 3 Department of Thoracic Surgery, Huashan Hospital, Fudan University, Shanghai 200032, China; 4 Department of Thoracic Surgery, Shanghai Pulmonary Hospital, Tongji University, Shanghai 200433, China

## Abstract

Dysregulation of miRNAs is reported to be involved in the invasion and metastasis of lung cancer. Previous studies showed that low serum miR-499 expression was associated with advanced TNM stage and poor prognosis. The present study is carried out to evaluate the biological functions of miR-499-5p in lung cancer. We demonstrated that miR-499-5p was significantly reduced in NSCLC tissues and correlated with poor clinical outcomes. Overexpression of miR-499-5p inhibited cell proliferation and induced apoptosis *in vitro* and *in vivo*. Furthermore, miR-499-5p overexpression also inhibited NSCLC metastasis *in vitro* and *in vivo*. Using bioinformatics tools, we identified VAV3 as a candidate target of miR-499-5p, and demonstrated that restoration of miR-499-5p expression in NSCLC cells downregulated VAV3 expression while inhibition of miR-499-5p upregulated VAV3 expression. Luciferase reporter assays showed that miR-499-5p targeted 3′-UTR of VAV3. Moreover, cancer growth, proliferation and metastasis were decreased and apoptosis was increased after VAV3 blockage induced by miR-499-5p overexpression. We conclude that miR-499-5p functions as a tumor suppressor by targeting VAV3. This finding may provide a therapeutic approach for future treatment of NSCLC.

Lung cancer is the leading cause of cancer-related mortality, resulting in approximately 224,210 new cases and 159,260 deaths within the United States in 2014^1^. Non-small cell lung cancer (NSCLC) represents approximately 85% of all lung cancers, and is often discovered at the locally advanced or metastatic stage of the disease^2^. Despite improvements in targeted therapies including epithelial growth factor receptor (EGFR) targeting therapies, the 5-year overall survival (OS) rate of NSCLC patients is about 17%^3^. Thus, further investigation of the molecular mechanisms underlying the carcinogenesis and tumor progression is essential for developing new effective therapeutic targets and anti-lung cancer strategies. Accumulating evidence has shown that microRNAs (miRNAs) plays an important role in NSCLC pathogenesis, which provides novel insights into the treatment of lung cancer^4^.

miRNAs are a group of non-coding small RNAs (approximately 21–23 nucleotides in length) that can target multiple distinct transcripts, thus playing an important role in regulation of mRNA expression^5^. Several recent studies^6^,^7^ have also shown that dysregulation of miRNAs is involved in the initiation and progression of cancer. With an increased understanding about miRNA target genes and cellular mechanisms, miRNA function modulation may provide new opportunities for lung cancer therapy^8^.

Some previous studies^9^ reported that miR-499-5p promoted invasion and metastasis of colorectal cancer and might be a new potential therapeutic target for colorectal cancer. Hu *et al.*^10^ reported a four-miRNA signature (miR-486, miR-30d, miR-1 and miR-499) that predicted survival of stage I-IIIa NSCLC. Our previous study^11^ also showed that low serum miR-499 expression was associated with an advanced TNM stage and poor prognosis. However, there is limited evidence of miR-499-5p dysregulation in lung cancer and the detailed mechanism of the involvement and targets in lung cancer progression remain unclear.

The present study is carried out to extend our previous findings through identification of target genes for miR-499-5p, and evaluate its biological functions in lung cancer. We demonstrated that miR-499-5p inhibited NSCLC growth by suppressing cell proliferation and inducing apoptosis. Furthermore, the overexpression of miR-499-5p inhibited NSCLC metastasis. Our findings suggest that miR-499-5p may function as a tumor suppressor by directly targeting VAV-3.

## Results

### miR-499-5p is significantly reduced in NSCLC tissues and correlated with poor clinical outcomes

Our previous study^11^ demonstrated that the expression of miR-499-5p was significantly decreased in human NSCLC tissues compared with their matched normal lung tissues. It was found in the present study that the expression of miR-499-5p in tumor tissues was inversely associated with tumor and lymph node metastasis in NSCLC patients (Table 1). Kaplan-Meier analysis showed that the OS rate in NSCLC patients with low miR-499-5p levels was significantly lower than that in those with high miR-499-5p levels (P = 0.028, log-rank test, Fig. 1A). The multivariable Cox proportional hazards model showed that miR-499-5p was an independent predictor of prognosis in NSCLC patients (Table 2). These results suggest that miR-499-5p may be closely related to the progression and metastasis of NSCLC.

### miR-499-5p overexpression inhibits cell proliferation and induces apoptosis *in vitro* and *in vivo*

Lower expression of miR-499-5p was detected in NSCLC cell lines (A549, H23, H522 and HOP62) compared with human bronchial epithelial cells (BEAS-2B) (Fig. S1A). To investigate the potential role of miR-499-5p in regulating NSCLC cell growth, we overexpressed or inhibited miR-499-5p in several NSCLC cell lines. As shown in Fig. 1B, overexpression of miR-499-5p significantly inhibited NSCLC cell growth. In contrast, inhibition of miR-499-5p significantly promoted cell growth. These results were further confirmed by the clonogenic assay. As shown in Fig. 1C, overexpression or depletion of miR-499-5p inhibited or stimulated colony formation in NSCLC cells, respectively. BrdU analysis further confirmed that overexpressed or inhibited miR-499-5p suppressed or stimulated cell proliferation, respectively (Fig. S2). After that, the effect of miR-499-5p on NSCLC growth *in vivo* was evaluated in mouse xenograft models. We prepared stable miR-499-5p-expressing transfectants using a lentivirus system. Consistent results were also obtained from the *in vitro* experiments (Fig. 1D,E). Overexpressed or inhibited miR-499-5p suppressed or stimulated tumor growth, respectively. We also analyzed the cell cycle distributions of miR-499-5p or NC stably transfected-A549 and H23 cells to explain the cell growth suppression caused by miR-499-5p overexpression. As shown in Fig. S3, a significant increase in S-phase of cells from miR-499-5p overexpressing A549 and H23 cells was observed compared with those from NC-transfected cells. The data above indicated that miR-499-5p inhibited cell cycle progression through S-phase.

Additionally, the effect of miR-499-5p on NSCLC cell proliferation and apoptosis was further examined. As shown in Fig. 2A,B, overexpression or depletion of miR-499-5p significantly inhibited or stimulated cell proliferation, respectively. Furthermore, we found that A549 and H23 cells transfected with pre-miR-499 or miR-499-5p mimic showed an inhibited proliferation compared with those transfected with miR-499-3p mimic or control (Fig. S4). Meanwhile, apoptosis was induced or inhibited by overexpression or depletion of miR-499-5p, respectively. These results were confirmed in an A549 xenograft model. The level of Ki67 was significantly decreased in the miR-499-5p-overexpression xenograft model, and increased in the miR-499-5p-depletion model (Fig. 2C). Moreover, we evaluated the expression of cleaved PARP and caspase-3 in tumor tissues from the xenograft model. Caspase-3 was increased in the miR-499-5p-overexpression model and decreased in the miR-499-5p-depletion model (Fig. 2D). The above results indicate that miR-499-5p was a tumor suppressor in NSCLC cells.

### Overexpression of miR-499-5p inhibits NSCLC metastasis *in vitro* and *in vivo*

To further investigate the role of miR-499-5p involved in NSCLC metastasis, we performed the following studies. Western blotting results showed that the expression of E-cadherin was increased and that of vimentin was decreased significantly in miR-499-5p overexpression A549 cells (Fig. 3A). Conversely, reduced E-cadherin and increased vimentin were detected in miR-499-5p inhibition H23 cells (Fig. 3A). Consistent results were also obtained using IF analysis (Fig. 3B). To examine the correlation between miR-499-5p expression and extracellular matrix (ECM) degradation, western blotting analysis was performed. As shown in Fig. S5A, protein expression level of MMP-2, MMP-9 in A549 and H23 cells was not changed by miR-499-5p and miR-499-5p inhibitor. Moreover, we demonstrated that the expression of E-cadherin and vimentin was not markedly changed by VAV3 in A549 cells (Fig. S5B). In addition, we also found that cell invasion was suppressed or stimulated when miR-499-5p was overexpressed or inhibited (Fig. 3C). The transfection efficiency was estimated by qRT-PCR (Fig. S6).

In addition, we used an A549 xenograft model to evaluated the effect of miR-499-5p dysregulated expression on NSCLC metastasis. NSCLC cells stably expressing miR-499-5p or antisense miR-499-5p was injected into the nude mice through the tail vein. As expected, miR-499-5p suppressed lung metastasis formation. The number of lung metastatic nodules was significantly decreased in the miR-499-5p overexpression group and increased in the miR-499-5p inhibitor group compared with the control group (Fig. 3D). These observations indicate that miR-499-5p is a negative regulator of NSCLC metastasis.

### miR-499-5p inhibits NSCLC cell growth and metastasis by directly targeting VAV3

To clarify the molecular mechanisms of miR-499-5p on the metastasis of NSCLC cells, we searched for the target genes using TargetScan and miRanda. VAV3 was identified as one of the candidate targets of miR-499-5p, based on putative target sequences at 383–389 and 142–149 bp of VAV3. The sequences were conserved in different species, as shown in Fig. 4A. Overexpression of miR-499-5p decreased the VAV3 expression, while inhibition of miR-499-5p increased VAV3 expression at both mRNA and protein levels (Fig. 4B,C). To confirm the prediction, we performed luciferase reporter assay. As indicated in Fig. S7, we inserted a three-nucleotide mutation into the 3′-UTRs of VAV3 and the corresponding mutant counterparts were also inserted into the luciferase reporter gene. As shown in Fig. 4D, miR-499-5p reduced the luciferase activity of VAV3 with the wild-type 3′-UTR, and the suppressive effect was significantly reversed in VAV3 with mutant miR-499-5p target sequences in A549 cells. Inverse correlation of miR-499-5p and VAV3 mRNA was also observed in A549 and H23 cells (Fig. S1B). In addition, the expression of miR-499-5p was inversely correlated with VAV3 expression in NSCLC patient specimens (Fig. 4E). VAV3 expression levels were much higher in patients with low miR-499-5p expression than those in patients with high expression (Fig. 4E). Furthermore, NSCLC patients with high VAV3 levels had significantly shorter OS compared with those with low VAV3 levels (*p* = 0.02, Fig. 5F). In conclusion, these data suggest that miR-499-5p negatively regulates the expression of VAV3 by directly targeting their 3′-UTR sequences.

To see whether VAV3 overexpression contributed to cell growth and metastasis, we overexpressed VAV3 in miR-499-5p-overexpression A549 cells. As shown in Fig. 5, exogenous overexpression of VAV3 in A549 significantly blocked the induction of apoptosis and inhibition of cell proliferation and metastasis by miR-499-5p. These data indicate that VAV3 plays an important role in the effects of miR-499-5p on NSCLC cell growth and metastasis.

## Discussion

Recently, miRNAs have been shown to regulate gene and protein expression and be involved in lung cancer progression and metastasis^12^. Previous evidence has indicated that miR-499-5p promoted metastasis of CRC cells and lower serum miR-499-5p is confirmed in NSCLC patients and associated with shorter OS^9^,^11^. It was found in our previous work^11^ that serum miR-499 levels were decreased in NSCLC patients compared with control subjects. Lower serum miR-499 levels were associated with poorer OS and considered as an independent prognostic marker in NSCLC patients. In addition, lower serum miR-499 levels in stage I-II NSCLC patients showed a shorter disease-free survival (DFS). Although miR-499-5p is shown to be involved in various heart diseases^13^, little is known about miR-499-5p involvement in lung tumorigenesis.

In the present study, we investigated the precise biological role of miR-499-5p expression in NSCLC. It was found that the expression level of miR-499-5p was downregulated in NSCLC tissues and inversely correlated with NSCLC metastasis and clinical stages. Moreover, lower miR-499-5p level might be correlated with shorter OS survival in NSCLC patients. These results suggest that miR-499-5p level in the tumor tissue is closely related to the progression and metastasis of NSCLC. Furthermore, we investigated the effect of miR-499-5p on NSCLC growth and found that miR-499-5p played an important role in NSCLC growth. In our study, we demonstrated that miR-499-5p overexpression inhibited NSCLC cells proliferation, induced cell cycle arrest and apoptosis. After that, we focused on the effect of miR-499-5p on NSCLC metastasis. Western blotting and IF analysis showed that E-cadherin was reduced and vimentin was increased in miR-499-5p inhibition cells. We also found that cell invasion was suppressed when miR-499-5p was overexpressed. The A549 xenograft model showed that the number of lung metastatic nodules was decreased in miR-499-5p overexpression group and increased in miR-499-5p inhibitor group. These observations indicate that miR-499-5p may act as a tumor suppressor during NSCLC metastasis.

Additionally, we investigated the molecular mechanism and targets of miR-499-5p in NSCLC progression. Several bioinformatics tools were used to predict target genes of miR-499-5p, and VAV3 was identified to be a critical downstream target of miR-499-5p. VAV3, a guanine nucleotide exchange factor (GEF) for Rho GTPases, belongs to the subfamily of diffuse B-cell lymphoma GEF proteins that also includes VAV1 and VAV2^14^. VAV proteins are involved in a variety of cellular signaling processes including phagocytosis, cytoskeleton organization and cell transformation^15^. VAV3 mRNA was markedly increased in breast cancer specimens and regulated biological parameters critical for the growth of breast tumors and their metastatic dissemination to the lung^16^. In addition, VAV3 was reported to be directly correlated with tumor recurrence and overall patient survival^17^. VAV3 expression was also elevated in androgen refractile prostate cancer cell lines and prostate cancer clinical specimens^18^. VAV3 knockdown greatly attenuated prostate cancer cell proliferation^19^ and inhibited breast cancer cell growth^20^. VAV1 was associated with lung tumor size and played a critical role in the tumorigenicity of lung cancer cells^21^. However, the expression status and biologic function of VAV3 in lung cancer remain unclear.

In this study, we demonstrated that restoration of miR-499-5p expression in NSCLC cells downregulated VAV3 expression, while inhibition of miR-499-5p upregulated VAV3 expression. Luciferase reporter assays showed that miR-499-5p targeted the 3′-UTR of VAV3. Our data also indicate that cancer growth, proliferation and metastasis were decreased and apoptosis was increased after VAV3 blockage induced by miR-499-5p overexpression. In addition, the expression of miR-499-5p was inversely correlated with VAV3 expression in NSCLC patient specimens. Furthermore, clinical data showed that NSCLC patients with high VAV3 levels had significantly shorter OS. In conclusion, VAV3 played an important role in the effect of miR-499-5p on NSCLC cell growth and metastasis.

This is the first study to show that miR-499-5p significantly suppressed the NSCLC growth and metastasis *in vitro* and *in vivo* by targeting VAV3. In contrast to our results, Liu *et al.*^9^ demonstrated that miR-499-5p overexpression promoted cell migration and invasion in human colorectal cancer cell lines by targeting FOXO4 and PDCD4. However, our western blot analysis indicated that the overexpression of miR-499-5p did not alter the expression of FOXO4 and PDCD4 in A549 cells. Several studies^22^,^23^ also demonstrated that some special miRNA played different roles by targeting different genes in different cancers.

To investigate the mechanism underlying VAV3 regulation at the posttranscriptional level, we conducted a luciferase reporter test and found that miR-499-5p binding to the 3′-UTR of VAV3 decreased the expression of VAV3 at both mRNA and protein levels. However, the molecular mechanism of VAV3 involvement in NSCLC growth and metastasis remains unclear. Lin *et al.*^24^ indicated that VAV3 recruited upon activation of EphA2 and then promoted Rac1 activation to regulate invasion of prostate cancer cells. However, further experiments should be performed to detect the functional role of VAV3-Rac1 signaling pathway in NSCLC. Citterio *et al.*^16^ reported that VAV proteins control a large subset of cancer cell transcriptomes, including mRNA encoding proteins that play critical roles in both primary tumorigenesis and lung-specific metastasis in breast cancer cells. Therefore, our future research will focus on the specific mechanism underlying VAV3 involvement in NSCLC.

In summary, we have demonstrated that miR-499-5p functions as a tumor suppressor in NSCLC, and that VAV3 is a potential target of miR-499-5p in NSCLC. Although the mechanism underlying NSCLC progression remains elusive, our data may provide a strategy for targeting miR-499-5p as a novel therapeutic application for advanced NSCLC patients.

## Materials and Methods

### NNSCLC cancer tissue

This study was approved by the ethical review committee of Shanghai Pulmonary Hospital. All the experiments were performed in accordance with relevant guidelines and regulations. Frozen tumor specimens from 223 newly diagnosed NSCLC patients at Shanghai Pulmonary Hospital were analyzed for the expression of miR-499-5p. Primary tumor tissues were collected by surgical removal or biopsy and snap-frozen in liquid nitrogen until total RNA was extracted. Patients included were 32 to 81 years old and none received chemotherapy or radiotherapy before tissues collection. The patients’ characteristics are summarized in Table 1. This study was approved by the Institutional Review Board of Shanghai Pulmonary Hospital and informed consent was obtained from all patients.

### Total RNA extraction and quantitative RT-PCR analysis of miRNA

Total RNAs were extracted from the frozen tissue samples and cell lines with Trizol reagent (Invitrogen, USA). miRNAs were extracted using PureLink™ microRNA Isolation Kit (Life Technologies Corporation, Carlsbad, CA). Quantitative RT-PCR (qRT-PCR) for miR-499-5p, RNU6 and VAV-3 was performed in triplicate using the TaqMan microRNA Reverse Transcription Kit (Applied Biosystems, USA). qRT-PCR was performed in an ABI Prism 7000 sequence detection system (Applied Biosystems, USA) according to the manufacturer’s instructions, with the following cycling conditions: 94 °C for 10 min, followed by 40 cycles at 94 °C for 20s and 60 °C for 45s. miR-499 expression was calculated and normalized to RNU6 using the 2^–ΔΔCt^ method. All primers were synthesized by Sangon Biotech (Shanghai, China). The information of the primer sequences used was as follows: VAV3 (forward primer: 5′-TGAAGGCAGAGGAAGCACAT-3′ and reverse primer: 5′-GCATAGGAACCACAAGCAAGT-3′), β-Actin (forward primer: 5′-GTCATTCCAAATATGAGATGCGT-3′ and reverse primer: 5′-GCATTACATAATTTACACGAAAGCA-3′), RNU6 (forward primer: 5′–CTCGCTTCGGCAGCACA-3′ and reverse primer: 5′-AACGCTTCACGAATTTGCGT-3′).

### Identification of miR-499-5p target genes

Putative target genes of miR-499-5p were predicted using TargetScan (http://www.targetscan.org/) and miRanda (http://www.microrna.org/). To verify the precise target of miR-499-5p, the luciferase reporter assay was utilized.

### Western blot

Cell proteins were extracted and separated with sodium dodecyl sulfatepolyacrylamide polyacrylamide gel electrophoresis (SDS-PAGE), and transferred to a nitrocellulose filter membrane (Millipore, Billerica, MA) according to standard procedures. β-actin was used as a loading control. Antibodies were obtained from Univ-bio Inc (Shanghai, China). Band intensities were quantitated with ImageJ software (National Institutes of Health, Bethesda, MD).

### Immunofluorescence and immunohistochemic alanalysis

Immunohistochemical staining was performed to detect the expression of ki-67 in NSCLC tissues. Anti-ki-67 (Clone MIB-1, DAKO) was used as primary antibody. The immunohistochemical staining was evaluated based on a four-tier system that depended on positive staining for Ki-67. Immunohistochemical staining in NSCLC tissues were independently assessed and scored by two pathologists. For immunofluorescence assays, cells were transfected with the indicated oligonucleotides. Then transfected cells were seeded onto glass slides for 20 h and fixed with 4% paraforma ldehyde. The slides were then incubated with Anti-E-cadherin and Anti-N-cadherin (Cell Signaling Technology, Beverly, MA). Finally, the slides were incubated with fluorescence-labeled secondary antibody conjugates (Sigma1:50).

### Cell culture and transfection

Human NSCLC cell lines (A549, H23, H522 and HOP62) and human bronchial epithelial cells (BEAS-2B) were cultured in RPMI 1640 medium (GIBCO, Grand Island, NY) supplemented with 10% heat inactivated fetal bovine serum (FBS) and 1% penicillin–streptomycin at 37 °C in a humidified air atmosphere containing 5% CO_2_. Cells were transfected with the indicated nucleotides using lipofectamine 2000 (Invitrogen) according to the manufacturer’s directions. All plasmid vectors (pcDNA/miR-499-5p and empty vector) for transfection were extracted by DNA Midiprep or Midiprep kit (Qiagen, Hilden, Germany). miR-499-5p inhibitor and negative control oligonucleotide were synthesized by GenePharma, Shanghai, China.

### MTT and cell proliferation assay

After 4-h nucleotide transfection, cells were plated onto 96-well plates. The cell viability was measured using MTT according to the manufacturer’s protocol after being incubated with the indicated drug for 48 h. Cell proliferation was assessed in triplicate at indicated time points after transfection using Coulter counter according to the manufacturer’s instruction.

### BrdU incorporation assay

Immunocytofluorescence was performed on cells with anti-BrdU antibody and fluorochrome conjugated secondary antibody (YiBio, Shanghai, China). Nuclei were counterstained with 4′,6-diamidino-2-phenylindole (DAPI). Cells were analyzed under a fluorescent microscope. The immunohistochemically positive cells were then quantitatively expressed as a ratio to all DAPI-positive cells.

### Invasion and apoptosis analysis

Cells were transfected with indicated nucleotides for 24 h and 1 × 10^5^ cells in growth medium without serum were seeded in the upper wells of BD Chambers. The lower wells contained the same medium with 10% FBS. After 24 h, invading cells on the lower side of the chamber were fixed with 100% methanol for 10 min, air-dried, stained with 0.1% crystal violet, and counted. The assays were conducted three times independently. After 24-h transfection, cells were incubated with indicated drugs in culture plates. Twenty-four hours later, harvested cells were stained with annexin V and Propidium Iodide according to the manufacturer’s protocol.

### Cell cycle evaluation

Cells were fixed with 70% cold ethanol and incubated with fresh propidium iodide containing RNaseA for 30 min at 37 °C. A total of 10^4^ cells were analyzed by a FACS Calibur flow cytometer (Becton Dickinson, USA).

### Luciferase reporter assay

The precise target of miR-49-5p was verified using the Dual luciferase reporter assay system (Promega). Standard 3′- untranslated region (UTR) of VAV3 was amplified using PCR and cloned into a pGL3 vector. NSCLC cells (5 × 10^5^) were seeded in 24-well plates for 24 h, and then co-transfected with Luc-VAV3, Luc- VAV3-mu, or Luc-control vector. After two days, firefly and renilla luciferase activities were assayed using the Dual luciferase reporter assay system. Luciferase activities were normalized to Renilla luciferase. Experiments were performed three times in triplicate.

### *In vivo* tumor metastasis assay

The animal experiment was approved by the Animal Care and Use Committee at Shanghai 10^th^ People’s Hospital (Shanghai, China). Nude mice were purchased from Shanghai Laboratory Animal Center of China. Stably expressing miR-499-5p or miR-499-5p-antisense cells were used for generating the xenograft model. For the subcutaneous tumor growth assay, 4 × 10^6^ cells in 100 ml PBS were subcutaneously injected into nude mice (8 mice/group). All mice were sacrificed in 6 weeks, and the tumor weights were measured. For the intravenous injection assay, 5 × 10^6^ cells in 100 ml PBS were injected into the lateral tail vein of nude mice (8 mice/group). All mice were killed in 6 weeks, and metastatic nodules on the surface of the lung were counted.

### Statistical analysis

Data are presented as mean ± standard deviation (SD). Median expression of miR-499-5p and VAV3 was used as the cut-off point for high versus low level. Student’s t-test or one-way analysis of variance test (ANOVA) or chi-square test was used to assess the differences between the treatment groups. Kaplan-Meier survival analysis was used to estimate OS. Cox regression analysis was used to calculate univariate and multivariate hazard ratios for prognosis with a step-down method. Statistical tests were performed with Medcalc version 11.2 (Broekstraat 52, 9030; Mariakerke, Belgium). A value of P < 0.05 was defined as statistically significant.

## Additional Information

**How to cite this article**: Li, M. *et al.* Overexpression of miR-499-5p inhibits non-small cell lung cancer proliferation and metastasis by targeting VAV3. *Sci. Rep.* **6**, 23100; doi: 10.1038/srep23100 (2016).

## Supplementary Material

Supplementary Information

## Figures and Tables

**Figure 1:** miR-499-5p is correlated with poor prognosis of NSCLC patients and inhibits cells growth *in vitro* and *in vivo*. (**A**) Overall survival of NSCLC patients with low and high miR-499-5p expression. (**B**) Overexpression or inhibition of miR-499-5p significantly inhibited or stimulated NSCLC cells growth. (**C**) Overexpression or depletion of miR-499-5p inhibited or stimulated colony formation in A549 and H23 cells. (**D**) Expression of miR-499-5p was increased or decreased in cells stably expressing miR-499-5p or miR-499-5p-antisense compared to vector control. (**E**) Overexpression or inhibition of miR-499-5p inhibited tumor growth in A549 xenograft model or stimulated tumor growth in H23 xenograft model, respectively. Error bars represent the mean ± s.d. of three independent experiments. *p < 0.05; **p < 0.01; ***p < 0.001.

**Figure 2:** miR-499-5p inhibits cells proliferation and induces apoptosis *in vitro* and *in vivo*. (**A**) Overexpression or inhibition of miR-499-5p significantly arrested or accelerated NSCLC cell proliferation. (**B**) Overexpression or inhibition of miR-499-5p induced or inhibited apoptosis in HOP62 or H522 cells. (**C**) Expression of Ki-67 was decreased or increased by overexpression or inhibition of miR-499-5p in xenograft tumor samples. (**D**) Caspase-3 was increased or decreased by overexpression or inhibition of miR-499-5p xenograft samples. Error bars represent the mean ± s.d. of three independent experiments. *p < 0.05; **p < 0.01; ***p < 0.001.

**Figure 3:** miR-499-5p inhibits NSCLC metastasis *in vitro* and *in vivo*. (**A**) Western blot analysis shows miR-499-5p regulates E-cadherin and vimentin expression. (**B**) Immunofluorescence analysis of E-cadherin and vimentin expression in A549 cells transfected with miR-499-5p or miR-499-5p inhibitor. (**C**) miR-499-5p decreases HOP62 cells invasion, while inhibition of miR-499-5p increases H522 cells invasion. (**D**) The miR-499-5p or miR-499-5p inhibitors stably expressed cells were injected into the tail vein of nude mice. All mice were killed after six weeks, and the lung surface nodules were counted under microscopy. Error bars represent the mean ± s.d. of three independent experiments. *p < 0.05; **p < 0.01; ***p < 0.001.

**Figure 4:** miR-499-5p directly targets VAV3. (**A**) miR-499-5p target site resides at 383–389 of the VAV3 3′-UTR are conserved in different species. (**B**) VAV3 expression was negatively regulated by miR-499-5p at mRNA level. (**C**) Western blot analysis also showed miR-499-5p negatively regulated VAV3 expression. (**D**) Luciferase reporter assay for direct targeting of the 3′-UTR of VAV3 by miR-499-5p. Luciferase reporters with wild-type or mutant miR-499-5p target sequences of VAV3 were transfected into vector control or miR-499-5p stably infected A549 cells, and luciferase activity was measured according to the manufacturer’s protocol. (**E**) Inverse correlation of miR-499-5p and VAV3-protein was observed in NSCLC samples, and mRNA expression of VAV3 was high or low in low- or high-miR-499-5p human NSCLC samples. (**F**) Overall survival of NSCLC patients with low and high VAV3 expression. Error bars represent the mean ± s.d. of three independent experiments. *p < 0.05; **p < 0.01; ***p < 0.001.

**Figure 5:** VAV3 is involved in miR-499-5p-induced suppression of A549 cells growth, proliferation and invasion. (**A**) VAV3 blocked miR-499-5p induced inhibition of A549 cell colony formation. (**B**) VAV3 blocked miR-499-5p induced A549 cell proliferation inhibition. (**C**) VAV3 blocked inhibition of A549 cells invasion by miR-499-5p. (**D**) VAV3 blocked miR-499-5p induced A549 cells apoptosis. Error bars represent the mean ± s.d. of three independent experiments. *p < 0.05; **p < 0.01; ***p < 0.001.

**Table 1:** Association between miR-499-5p expression in tissue and patients’characteristics.

Factors	Tissue miR-499-5p (n = 223)		*P*
	Low (n = 112)	High (n = 111)	
Age (years)			0.17
≤65	27	37	
>65	85	74	
Gender			0.35
Male	60	52	
Female	52	60	
Smoking status			0.84
Nonsmoker	58	55	
Ever-smoker	54	56	
Histologic type			0.52
Adenocarcinoma	40	43	
Squamous	62	54	
Others	10	14	
T status			<0.001
T1	26	52	
T2	51	46	
T3	6	4	
T4	28	10	
N status			0.001
N0	60	74	
N1	20	25	
N2	22	5	
N3	10	4	
M status			<0.001
M0	90	107	
M1a	10	1	
M1b	12	3	
EGFR mutation status			0.25
Mutated	41	50	
Wild type	71	61	

EGFR, epidermal growth factor receptor.

**Table 2:** Univariate and multivariate analyses for prognostic factors in patients with NSCLC.

Variables	Univariate			Multivariate		
	HR	95% CI	*P*	HR	95% CI	*P*
**Age, years (>65 vs ≤ 65)**	0.75	0.51–1.09	0.11	—	—	—
**Gender (female vs male)**	1.18	0.83–1.69	0.34	—	—	—
**Histology (squamous vs non-squamous)**	1.21	0.85–1.72	0.29	—	—	—
**Pathological T (T3/4 vs T1/2)**	2.14	1.42–3.22	<0.001	1.60	1.04–2.47	0.03
**Lymph node metastasis (N1-3 vs N0)**	1.96	1.32–2.90	0.001	1.31	1.02–1.68	0.03
**Distant Metastasis (M1 vs M0)**	5.06	2.33–11.00	<0.001	3.72	2.19–6.34	<0.001
**miR-499-5p in tumor (high vs low)**	0.68	0.48–0.97	0.028	0.65	0.45–0.95	0.027
**EGFR status (Mutation vs Wild type)**	0.96	0.68–1.37	0.83	—	—	—

HR, hazard ratio; CI, confidence interval; EGFR, epidermal growth factor receptor.
